The article "Clinical significance of serum MicroRNA-203 in patients with acute myeloid leukemia" was retracted in 2020. Reasons: plagiarism; overlap with other authors' work.

# Clinical significance of serum MicroRNA-203 in patients with acute myeloid leukemia

**DOI:** 10.1080/21655979.2019.1652490

**Published:** 2019-08-14

**Authors:** Yingmeng Guo

**Affiliations:** Department of Pediatric medicine, Linyi Central Hospital, Yishui, China

**Keywords:** serum miR-203, acute myeloid leukemia, diagnosis, prognosis

## Abstract

This study aimed to detect serum miR-203 expression levels in AML and explore its potential clinical significance. Quantitative reverse transcriptase polymerase chain reaction (qRT-PCR) was performed to measure the serum miR-203 levels in 134 patients with AML and 70 healthy controls. The results demonstrated that serum miR-203 expression was significantly reduced in AML patients compared with healthy controls. Receiver operating characteristic curve (ROC) analysis revealed miR-203 could distinguish AML cases from normal controls. Low serum miR-203 levels were associated with worse clinical features, as well as poorer overall survival and relapse free survival of AML patients. Moreover, multivariate analysis confirmed low serum miR-203 expression to be an independent unfavorable prognostic predictor for AML. The bioinformatics analysis showed that the downstream genes and pathways of miR-203 was closely associated with tumorigenesis. Downregulation of miR-203 in AML cell lines upregulated the expression levels of oncogenic promoters such as CREB1, SRC and HDAC1. Thus, these findings demonstrated that serum miR-203 might be a promising biomarker for the diagnosis and prognosis of AML.

## Introduction

Acute myeloid leukemia (AML) is an aggressive, heterogeneous, myeloid malignancy characterized by the abnormal proliferation and differentiation of myeloid progenitor cells [1]; in 2018 an estimated 19,520 new cases and 10,670 deaths occurred in the US [2]. Despite a growing list of treatment options, most patients still relapse and die after remission, and the prognosis remains unideal [3]. It is necessary to explore new biomarkers for diagnosis, prognostication, and therapeutic targets of AML so as to develop more effective surveillance and treatment programs.

MicroRNAs (miRNAs) are evolutionary conserved short non-coding single-stranded RNAs (19–22 nucleotides) that negatively regulate mRNA stability [4]. They play an essential role in many biological functions, such as cell growth, proliferation, differentiation, and apoptosis [5]. Moreover, miRNAs can act as oncogenes or tumor suppressors, contributing to malignant transformation in solid and hematological tumors, including AML [6,7]. In addition, miRNAs regulate different mRNA targets, and their modulation can represent a potential therapeutic target in leukemic progenitors, as well as in leukemia stem cells (LSCs).

miRNAs have many properties of good AML prognostic biomarkers, such as wide presence in various tissues, highly conserved sequences, and easy and sensitive detection, as well as stability under extreme conditions [8]. Mounting studies have shown that miRNAs can be used to predict outcome in CN-AML. Zhang et al. reported miR-216b overexpression as an independently poor prognostic factor for CN-AML and may provide a valuable biomarker associated with disease recurrence in AML [9]. In 224 patients with CN-AML, high miR-362-5p expression was associated with older age and shorter OS compared with low expressers [10]. Diaz-Beya et al. reported that high miR-3151 expression was commonly found in AML patients and obtained shorter disease-free, OS, lower CR rate and higher cumulative incidence of relapse compared with low expressers [11]. Several studies have reported that miR-203 functions as a tumor suppressor in various cancers, including leukemia, esophageal cancer, and breast cancer [12,13], inhibiting cancer cell proliferation [14]. MicroRNA-203 may also be a diagnostic and prognostic marker in patients with cancers, such as multiple myeloma [15], gastric cancer [16] and glioblastoma [17]. However, the clinical significance of serum miR- 203 in AML remains uncertain. In this study, we investigate serum miR-203 levels in AML patients and assess its potential clinical significance.

The article "Clinical significance of serum MicroRNA-203 in patients with acute myeloid leukemia" was retracted in 2020. Reasons: plagiarism; overlap with other authors' work.

## Materials and methods

### Cell culture and transfections

The AML cell lines THP-1 and K-562 were obtained from the American Type Culture Collection (ATCC, Manassas, VA, USA). and cultured in RPMI-1640 (GibcoR; Life Technologies, Carlsbad, CA, USA) supplemented with 10% fetal bovine serum (Invitrogen, Carlsbad, CA, USA). The miR-203 inhibitor and non-targeting control (scrambled miRNA) was procured from Ambion (Ambion, Austin, TX, USA). Lipofectamine RNAiMAX (Invitrogen, Carlsbad, CA,USA) was used to transfect AML cells with 50 nmol/L of the miR- 203 inhibitor or scrambled miRNA based on the manufacturer’s instructions.

### Patient samples

The study was approved by the Ethics Committee of Linyi central Hospital. A total of 134 cases diagnosed with de novo AML (non-M3) were enrolled. According to the French-America-British (FAB) classification, 7 patients had AML M0, 40 had M1, 52 had M2, 17 had M4, 15 had M5, and 3 had M7. 70 healthy volunteers was recruited as the controls and none of them had any clinical symptoms of cancer or other diseases. AML complete remission (CR) was defined as a normocellular BM containing less than 5% blasts and normalization of the peripheral blood counts at one month after starting induction therapy. Prior informed consent was obtained from all participants. Up to 5 ml whole blood was withdrawn from each participant and collected in EDTA-K2 tubes. Subsequently, the supernatant was isolated from blood samples by centrifuging at 1200 g for 10 min, then centrifuged at 12,000 g for 10 min at 4°C, and transferred to cryotubes and stored at −80°C.

The article "Clinical significance of serum MicroRNA-203 in patients with acute myeloid leukemia" was retracted in 2020. Reasons: plagiarism; overlap with other authors' work.

### RNA extraction, quantitative reverse transcriptase polymerase chain reaction (qRT-PCR)

Total RNA was extracted from the serum using a QIAamp RNA Blood kit (Qiagen, Hilden, Germany) in accordance with the manufacturer’s protocols. The quantity and concentration of RNA were spectrophotometrically assessed by measuring absorbance at A260/280. Reverse transcription reactions were carried out with the Prime-Script RT reagent kit (TaKaRa, Dalian, China). Quantitative RT-PCR was run on an ABI 7500 Real-Time PCR System (Applied Biosystems, Foster City, CA, USA) using miScript SYBR green PCR kit (Qiagen, Hilden, Germany). The relative miR-203 expression was calculated by the comparative 2-ΔΔCt method using cer-miR-39 as the endogenous control. Triplicates were performed for all qRT-PCR reactions. Bioinformatic analysis of the downstream genes of miR-203 The targeted genes of miR-203 were obtained from TargetScan7.2 (http://www.targetscan. org/vert_71/). Gene Ontology (GO) and Kyoto Encyclopedia of Genes and Genomes (KEGG) pathway enrichment analyses were performed using the Database for Annotation, Visualization and Integrated Discovery (DAVID) database (https://david.ncifcrf.gov/). STRING online database (https://string-db.org/) was used for the protein-protein interaction (PPI) analysis. The central nodes with most connections were chosen for validation in AML cell lines.

### Statistical analysis

All statistical analyses were performed using Student GraphPad Prism 5 (GraphPad Software, Inc., La Jolla, CA, USA). Overall survival (OS) was defined as the time from diagnosis of AML to any cause of death. Relapse-free survival (RFS) was defined as the time from CR to relapse or death. The Mann-Whitney U test or KruskalWallis test were used to assess a significant difference in serum miR-203 expression between two groups or among multiple groups respectively. Chi-square analysis was used to evaluate the difference of categorical variables. The receiver operating characteristic (ROC) curve was constructed to determine the diagnosis value of serum miR-203 level. KaplanMeier method was used to estimate the relationship between miR-203 expression and OS and RFS. Multivariate survival analysis was performed using the Cox proportional hazards model. Differences were considered statistically significant when P < 0.05.

The article "Clinical significance of serum MicroRNA-203 in patients with acute myeloid leukemia" was retracted in 2020. Reasons: plagiarism; overlap with other authors' work.

## Results

### Reduced serum miR-203 expression in AML patients

miR-203 levels were detected in blood samples from all participants by qRT-PCR assay. As shown in Figure 1(a), serum miR-203 expression was 0.46 ± 0.17 in AML patients, which was greatly decreased compared to that in healthy controls (0.71 ± 0.23) (*P* < 0.05). The serum miR-203 expression was 0.27 ± 0.09, 0.41 ± 0.13, 0.49 ± 0.12, 0.53 ± 0.16, 0.51 ± 0.14, 0.39 ± 0.11 in AML subtypes M0, M1, M2, M4, M5 and M7,respectively, which was greatly decreased compared to that in healthy controls (*P* < 0.05). No significant difference was observed in serum miR-203 expression among AML subtypes (P > 0.05, Figure 1(b)).

**Figure 1.** Serum miR-203 was detected by qRT-PCR in patients and health controls. (a). Serum miR-203 expression in blood samples. Plots depicting the relative expression for blood levels of miR-203 between AML patients and healthy controls. (b), Serum miR-203 expression in blood samples in different AML subtypes. *P < 0.05.

### The diagnostic value of serum miR-203 for AML

ROC curve analysis identified serum miR-203 expression as a reliable biomarker for discriminating AML subjects from controls with the area under the ROC curve (AUC) of 0.853, and the sensitivity and specificity were 77.61% and 81.43%, respectively (Figure 2). Among all AML patients, 57 cases achieved CR. We compared the miR- 203 levels in paired blood samples of these patients and found miR-203 expression was significantly upregulated when CR was achieved after chemotherapy (P < 0.05,Figure 3).

**Figure 2.** The role of blood miR-203 in AML diagnosis using Receiver-operating characteristic (ROC) curve analysis.

**Figure 3.** Comparison of miR-203 levels in 57 paired serum samples before and after CR.

### Correlation between serum miR-203 expression and clinicopathologic factors

The AML patients were divided into high and low serum miR-203 expression group based on the median fold-change values. Serum miR-203 expression was significantly associated with cytogenetics (P = 0.0166), complete remission (P = 0.0178), and FAB classification (P = 0.0039). However, other clinical characteristics including gender, age, bone marrow blasts and white blood cells (WBC) were not directly correlated to serum miR-203 expression.

### Correlation between serum miR-203 expression and prognosis of AML

Kaplan-Meier analysis revealed that AML patients with low serum miR-203 levels had shorter OS and RFS rates than those with high serum miR-203 levels (P = 0.016, Figure 4(a); P = 0.012, Figure 4(b), respectively). Multivariate survival analysis demonstrated that serum miR-203 level (OS: OR = 3.35, 95% CI = 1.78–5.06, P = 0.002; RFS: OR = 3.02, 95% CI = 1.52–4.73, P = 0.003), cytogenetics (OS: OR = 2.67, 95% CI = 1.34–4.15, P = 0.005; RFS: OR = 2.27, 95% CI = 1.07–3.55, P = 0.008), and FAB classification (OS: OR = 2.86, 95% CI = 1.43–4.35, P = 0.004; RFS: OR = 2.36, 95% CI = 1.14–3.69, P = 0.008) were prognostic markers for OS and RFS.

The article "Clinical significance of serum MicroRNA-203 in patients with acute myeloid leukemia" was retracted in 2020. Reasons: plagiarism; overlap with other authors' work.

**Figure 4.** Serum miR-203 expression levels are associated with poor prognosis in AML patients. (a), Kaplan-Meier curve showing the overall survival (OS) of patients with high and low miR-203 expression. (b), Kaplan-Meier curve showing the progression-free survival (PFS) of patients with high and low miR-203 expression.

### Bioinformatics analysis

Bioinformatic analysis showed that GO:00–45,893~positive regulation of transcription, DNA-templated, GO:0045944~positive regulation of transcription from RNA polymerase II promoter and GO:0000122~negative regulation of transcription from RNA polymerase II promoter were the top biologic processes. GO:0005634~nucleus, GO:0005654~nucleoplasm, GO:0005737~cytoplasm, were the top enriched cellular components. GO:0001077~transcritional activator activity, RNA polymerase II core promoter proximal region sequencespecific binding, GO:0005515~protein binding and GO:0043565~sequence-specific DNA binding were the top enriched in molecular function. TGF-beta signaling pathway, FoxO signaling pathway, Signaling pathways regulating pluripotency of stem cells, Wnt signaling pathway, and Insulin signaling pathway were the top enriched KEGG pathways (Figure 5). We first identified the central nodes of the PPI network from the downstream targets (connections ≥20) (Figure 6(a)). Our qPCR results showed that the expression levels of CREB1, SRC, and HDAC1 were significantly higher in AML cell lines subjected to miR-203 inhibitor transfection compared to the controls (Figure 6(b)).

**Figure 5.** The downstream genes of miR-203 were detected by GO and KEGG analysis.

**Figure 6.** Effect of targeting miR-203 on the downstreams of miR-203. (a), The central nodes of the PPI network. (b), The expression levels of CREB1, SRC and HDAC1 were significantly higher in AML cells subjected to miR-203 suppression.

## Discussion

The current gold standard of cancer diagnosis is the histological examination of tissue, obtained either by radiologically guided biopsy or surgical excision. However, these procedures are invasive, expensive, and not without risk to the patient. They also take time and need to be consistently evaluated by expert pathologists. Therefore, there is a clear clinical need for alternative diagnostic techniques. In particular, the use of biological fluids such as blood as a source of non-invasive biomarkers of cancer has raised a great deal of interest [18]. An ideal biomarker should have a high specificity, sensitivity, and predictive power. miRNAs have a number of intrinsic characteristics that make them attractive as biomarkers. Firstly, they are highly specific, and it has been shown that miRNA expression profiles differ between cancer types according to diagnosis and the developmental stage of the tumor, with a greater resolution than traditional gene expression analysis [19]. Secondly, unlike other RNA classes, miRNAs are remarkably stable and therefore can be robustly measured not only in biological fluids but also from routinely prepared formalin-fixed paraffin-embedded (FFPE) material [14].

miR-203 is one of the most studied miRNAs to be a potential biomarker for diagnosis and prognosis of cervical cancer [20], esophageal squamous cell carcinoma [21], gastric cancer [15] and colorectal cancer [22]. Zhang et al verified that deletion of serum miR-203 was found in patients with bladder cancer, and reduced serum miR-203 predicted poorer survival [23]. In gastric cancer, Chu and colleagues reported that low miR-203 expression predicted poor prognosis of patients [24]. Our study demonstrated that serum miR-203 was significantly lower in AML patients and AML patients with low serum miR-203 had shorter survival, and serum miR-203 was an independent indicator of OS/RFS by multivariate analysis. In addition, serum miR-203 was closely associated with cytogenetics, complete remission and FAB classification and serum miR-203 was a potential marker for diagnosis of AML.

miR-203 had been reported to exert a tumor suppressive role in multiple cancers through its downstreams. For instance, miR-203 induced apoptosis of bladder cancer cells in vitro and in vivo by bcl-w downregulation [25]. Ectopic expression of miR-203 suppressed bladder cancer tumorigenic potential and enhanced cisplatin cytotoxicity by regulating Bcl-w and survivin [23]. In lung cancer, overexpression of miR-203 greatly reduced cancer cell proliferation, and migration and stimulated apoptosis via degrading LIN28B [26], PKCα [26] and SRC [27]. In osteosarcoma, miR-203 markedly inhibited cancer cell growth, invasion, migration, and suppressed mesenchymal-toepithelial reversion transition (MErT) through targeting RAB22A or TBK1 [28,29]. In cervical cancer cells, miR-203 greatly suppressed tumorigenicity and angiogenesis in vivo by silencing VEGFA expression [30]. Miao et al revealed elevated miR-203 expression repressed cancer cell migration, invasion and epithelial to mesenchymal transition by targeting caveolin-1 in pancreatic cancer [31]. However, Greither and colleagues demonstrated high miR-203 expression was an independent indicator of shorter survival in patients with pancreatic ductal adenocarcinomas, indicating miR-203 might be an oncogenic miRNA [32]. Therefore, miR-203 might have different regulatory roles during the initiation and progression in some kinds of tumors. In our study, downregulation of miR-203 in AML cell lines upregulated the oncogenic promoters such as CREB1, SRC and HDAC1. Bioinformatics analysis showed that the downstream genes of miR-203 were closely associated with tumorigenesis. These results suggested that low serum miR-203 is an adverse prognostic factor in AML and might serve as a useful diagnostic and prognostic biomarker. However, the limitation of this study is the small sample size, and our results require further validation with large cohorts.

The article "Clinical significance of serum MicroRNA-203 in patients with acute myeloid leukemia" was retracted in 2020. Reasons: plagiarism; overlap with other authors' work.

## Conclusion

It has demonstrated that low serum miR-203 expression is associated with aggressive clinical features and poor survival in patients with AML. Serum miR-203 might be a promising marker for the diagnosis and prognosis of AML, and miR-203 might be a useful target for AML treatment.

## Highlights

1. Low serum miR-203 expression was detected in AML patient.
2. Low serum miR-203 expression was associated with poor prognosis in AML patient.
3. Serum miR-203 expression could discriminat AML patients from healthy controls with high sensitivity and specificity.
4. Targeting miR-203 in AML cell lines upregulated oncogenic promoters.
